# KIAA0101, a target gene of miR-429, enhances migration and chemoresistance of epithelial ovarian cancer cells

**DOI:** 10.1186/s12935-016-0353-y

**Published:** 2016-09-26

**Authors:** Hong Chen, Bairong Xia, Tianbo Liu, Mei Lin, Ge Lou

**Affiliations:** Department of Gynecology, the Affiliated Tumor Hospital, Harbin Medical University, 150 Haping Rd, Harbin, 150020 Heilongjiang China

**Keywords:** KIAA0101, miR-429, Epithelial ovarian cancer, Migration, Chemoresistance

## Abstract

**Background:**

Ovarian cancer is a common type of gynecological malignancies, and is the fifth leading cause of cancer-related death in women in the United States. MiR-429 and KIAA0101 have been found to be involved in several human malignancies, respectively. However, the role of miR-429 and KIAA0101, and the correlation between them during development of epithelial ovarian cancer (EOC) remain to be investigated.

**Methods:**

The expression of KIAA0101 in EOC tissues and cells was measured by Quantitative real-time PCR, western blot, and immunochemistry. Cell proliferation assay, colony formation assay, and transwell assay was performed to assess the role of miR-429 and KIAA0101 in regulation of proliferation, migration, and chemoresistance of EOC cells. Luciferase assay was used to test the Wnt/β-catenin signaling activity in response to depletion of KIAA0101 and overexpression of miR-429.

**Results:**

We found that KIAA0101 was upregulated in metastatic EOC tissues, compared to primary EOC tissues, and KIAA0101 was required for the migration activity and chemoresistance of EOC cells by enhancing Wnt/β-catenin signaling. Furthermore, we revealed KIAA0101 is direct target of miR-429. Similar to knockdown of KIAA0101, overexpression of miR-429 reduced invasion and chemoresistance of EOC cells. Co-transfection of KIAA0101 partially abrogates the inhibitory effects on invasion and chemoresistance in EOC cells.

**Conclusions:**

KIAA0101, a target gene of miR-429, was upregulated in the metastatic EOC tissues, and enhanced the migration activity and chemoresistance of EOC cells. Both miR-429 and KIAA0101 may represent the potential therapeutic targets of EOC.

## Background

Ovarian cancer is the one of the most lethal of gynecologic cancers, including epithelial ovarian cancer (EOC) [1, 2]. EOC is a common type of gynecological malignancy that accounts for the majority of gynecologic cancer-related, mainly because of the highly metastatic capacity of EOC cells [3]. During the progression of EOC, a portion of tumor cells may slough out from the primary sites, and subsequently spread throughout the peritoneal cavity [4, 5]. Due to the lack of reliable diagnostic biomarkers and the development of chemoresistance, the diagnosis and treatment of EOC remains to be a serious public challenge [6, 7]. Hence, it is crucial to improve our understanding in the underlying mechanisms that promotes metastasis and chemoresistance of EOC.

microRNAs (miRNAs) is a class of endogenous small non-coding RNAs, which are capable to post-transcriptionally modulate gene expression [8, 9]. In recent years, accumulating evidence has demonstrated that miRNAs are involved in cancer development by acting as oncogenes or tumor suppressors [9, 10]. MiR-429, a member of the miR-200 family of miRNAs, has been reported to inhibit invasion in gastric cancer [11], colorectal carcinoma [12], breast cancer [13], and oral squamous cell carcinoma [14], indicating a tumor suppressing effect of miR-429. However, higher expression of miR-429 was shown to be significantly correlated with a poor prognosis of patients with serous ovarian carcinoma (SOC) [15, 16]. These findings revealed different effects of miR-429 on cancer progression that are initiated from different tissues.

Proliferating cell nuclear antigen (PCNA) is an essential protein for DNA replication and repair, and high expression of PCNA is considered as a hallmark of cell proliferation, which is associated with high cell proliferation rate in cancers, such as prostate cancer and ovarian cancer [17]. KIAA0101, also known as p15PAF (PCNA-associate factor), contains a conserved PCNA-binding motif, and elevated KIAA0101 has been recently identified as an oncogene, and a potential biomarker for recurrence and poor prognosis in patients with lung cancer [18], esophageal cancer [19], and gastric cancer [20], respectively. Furthermore, overexpression of KIAA0101 during development of adrenal cancer was found to promote growth and invasion of tumor cells [21]. In addition, upregulation of KIAA0101 in patients with esophageal cancer was associated with progression and chemoresistance [19]. However, the role of KIAA0101 in regulation of development of EOC remains largely unknown. Specifically, the relationship between miR-429 and KIAA0101 is still unclear.

In this study, we examined the expression levels of miR-429 and KIAA0101 in primary and metastatic EOC tissues, and investigated the role of miR-429 and KIAA0101 in regulation of invasion and chemoresistance of EOCs. We found that miR-429 directly targeted the 3′ UTR of KIAA0101 transcripts, and negatively regulated the expression of KIAA0101. By using siRNA targeting KIAA0101, we demonstrated KIAA0101 is required for the invasion and chemoresistance to Cisplatin of EOC cells via promoting the translocation of β-catenin to nucleus. Finally, while overexpression of miR-429 exhibited an inhibition on invasion and chemoresistance, co-transfection of KIAA0101, at least in part, restored the invasion and chemoresistance of EOC cells.

## Methods

### Human samples

Tissues were collected from patients who underwent surgery at the Department of Obstetrics and Gynecology of Harbin Medical University Cancer Hospital between 2012 and 2013, including 40 epithelial EOC tissues and 20 normal epithelial ovarian tissue sections. None of the patients were treated with chemotherapy or radiotherapy before they were subjected to operation. The histopathological diagnoses were performed according to the World Health Organization criteria. All fresh specimens were stored at −80 °C for further use. This study was approved by the Medical Ethics Committee of Harbin Medical University Cancer Hospital and all patients were provided informed consent.

### Immunohistochemistry (IHC)

Tumor samples were fixed in 4 % formaldehyde, embedded in paraffin wax, and then cut into 5 µM sections. Samples were de-paraffinized in xylene and rehydrated. After blocking endogenous peroxidase and performing antigen retrieval, tissue slides were blocked in goat serum for 30 min and incubated with antibodies against KIAA0101 (1:100 dilution, Santa Cruz, Santa Cruz, CA, USA) overnight at 4 °C, followed by biotinylated secondary antibody (Santa Cruz) for 30 min. Staining was performed in parallel using a Vectastain ABC kit (Vector Laboratories, Burlingame, CA, USA).

### Cancer cell lines and culture

The human EOC cell lines SKOV3 and COV644 were supplied by China Center for Type Culture Collection (CCTCC). EOC cells were cultured in Dulbecco’s modified Eagle’s medium (DMEM; Gibco-BRL, Gaithersburg, MD, USA), supplemented with 10 % fetal bovine serum and antibiotics (Gibco). All cells were incubated at 37 °C under a humidified atmosphere containing 5 % CO_2_.

### Quantitative real-time PCR (qRT-PCR)

qRT-PCR was performed as previously described [22]. Briefly, total RNA was extracted using Trizol reagent (Invitrogen, Carlsbad, CA, USA). qRT-PCR analyses for mRNA of KIAA0101 were performed by using QIAGEN OneStep RT-PCR kits (Qiagen, Valencia, CA, USA). The mRNA level of β-actin was measured as an internal control. To measure miR-429 expression, total RNA was polyadenylated and reverse transcribed using TaqMan MicroRNA Reverse Transcription Kit and TaqMan miRNA assay (Applied Biosystems, Foster City, CA, USA) according to the manufacturer’s instructions. The expression of U6 small nuclear RNA was used as the internal control. RT-PCR was performed in triplicates. Relative expression of the tested genes was calculated and normalized using the 2^−ΔΔCt^ method. Primers were as follows: *KIAA0101* forward, 5′TCCTGAAGAGGCAGGAAGCAG T 3′, reverse, 5′ TTGTGTGATCAGGTTGCAAAGGA 3′; *β*-*actin* forward, 5′ TGACGGGGTCACCCACACTGTGCCCATCTA3′, reverse, 5′ CTAGAAGCATTTGCGGTGGACGATGGAGGG 3′.

### Transfection and luciferase assay

All oligonucleotides were transfected into EOC cells at a final concentration of 50 nM using HiPerFect transfection reagent according to the product manual (Qiagen). The wild type full-length 3′UTR of KIAA0101 gene containing the putative miR-429 biding sites was amplified by PCR and was inserted into the psiCHECK2 vector (Promega, Madison, WI, USA). The mutant KIAA0101 3′-UTR was generated from the KIAA0101 3′-UTR using the QuikChange^®^ Multi Site-Directed Mutagenesis kit (Stratagene, La Jolla, CA, USA). The coding sequences of KIAA0101 were generated by PCR and cloned into pCDNA3.1 (+) vector (Invitrogen) to generate pCDNA3.1-KIAA0101. The luciferase reporter vector (KIAA0101 3′UTR and TOP flash), pCDNA3.1-KIAA0101 and Renilla plasmid were all transfected using Lipofectamine LTX according to the manufacturer’s instructions.

Cells were seeded in triplicate in 24-well plates 1 day before transfection for the luciferase assay. 48 h after transfection, the cells were harvested and lysed, and the luciferase activity assayed using the dual-luciferase assay kit (Promega). Normalized luciferase activity was reported as luciferase activity/*Renilla* luciferase activity. Three independent experiments were performed.

### Cell proliferation assay

The cell growth rate with Cisplatin treatment were determined by MTT assay (Promega). Briefly, at 48 h after transfection, the cells were seeded into 96-well plates at 5000 per well in a final volume of 100 μl with different concentration of Cisplatin (0, 4, 8, 16, 32 and 64 µM). Then at 48 h, 25 µl of MTT stock solution was added to each well and incubated for 4 h. The absorbance was measured at 570 nM. The assays were performed in triplicate.

### Colony formation assay

The transfected EOC cells were seeded in 6-well plates (400 cells per well) and cultured for 10 days with different concentrations of Cisplatin (0, 8 and 32 µM). The cells were fixed with 10 % formalin, and stained with 0.5 % crystal violet (Sigma, St. Louis, MO, USA). The assay was performed in five replicates.

### Transwell migration and invasion assays

In vitro cell migration and invasion assays were performed using 24-well Transwell chambers (8-µM pores, BD Biosciences, San Jose, CA, USA). The transfected EOC cells (5 × 10^4^ cells per well) were cultured in the top chamber with 100 µl medium containing 1 % FBS. 500 μl complete media with 10 % FBS was added into the lower chamber. After 24 h of cultivation, the medium from the chamber and the Transwell were removed, and the chamber was gently wiped with a cotton swab. The migrated cells were fixed in 4 % paraformaldehyde, and stained with crystal violet solution. Six fields were randomly selected and counted. The procedure for the cell invasion assay was similar to the cell migration assay, except that the Transwell membranes were pre-coated with Matrigel (BD Biosciences). The assays were performed in triplicate.

### Western blot

Western blot was performed as described previously [23]. Briefly, Total protein was extracted by RIPA buffer. Nuclear protein was extracted using nuclear extracted kit (Beyotime, Beijing, China). The total extracts were separated using 10 % SDS–polyacrylamide gels and transferred onto polyvinylidene difluoride (PVDF) membranes (Bio-Rad, Hercules, CA, USA). The membranes were probed with a primary antibody against human KIAA0101, β-catenin, Axin2, c-myc, Histone or β-actin (Santa Cruz), respectively. After several washes with TBST, the membranes were incubated with (HRP)-conjugated secondary antibody (Santa Cruz). Bound antibody was detected using the Supersignal West Pico ECL chemiluminescence kit (Thermo scientific, Rockford, IL, USA).

### Statistical analysis

Statistical analyses were performed by SPSS Windows version 19. Data was expressed as mean ± SD of the experiments performed in triplicate. One-Way ANOVA was performed to determine the significance of difference among groups. Differences were considered significant at *p < 0.05, **p < 0.01 and ***p < 0.001.

## Results

### The expression of KIAA0101 is elevated in EOC samples

In order to determine the clinical relevance of KIAA0101 in human EOC development, we analyzed the expression levels of KIAA0101 in 40 primary EOC tumor tissues and 20 normal ovarian epithelial tissues. We found that compared to those in normal ovarian epithelial tissues, the levels of KIAA0101 expression were significantly higher in EOC tissues (Fig. 1a, *p* < 0.001). Cancer cells were found metastasized to the greater omentum in two of those EOC patients. Furthermore, we performed western blot to test KIAA0101 protein expression in primary EOC tissues and two EOC tissues with greater omentum, and found KIAA0101 was significantly higher in metastatic EOC tissues (Fig. 1b). Consistently, IHC results revealed that KIAA0101 staining was stronger in greater omentum metastatic EOC tissues compared to paired primary cancer tissues (Fig. 1c). Taken together, these data indicated that KIAA0101 was up-regulated in EOC tissues, and may play an important role in promoting EOC metastasis.

**Fig. 1:** Upregulation of KIAA0101 in ovarian cancer samples. **a** Relative mRNA levels of KIAA0101 was determined by qRT-PCR in 40 EOC tissues and in 20 normal epithelial tissues samples. *P* < 0.001. **b** KIAA0101 expression was determined by western blot in primary and greater omentum metastatic EOC tissues from two patients. **c** KIAA0101 expression was determined by IHC in primary and greater omentum metastatic EOC tissues. *Scale bar* 100 µM

### Knockdown of KIAA0101 inhibits EOC cell migration and invasion

Next, we sought to determine whether downregulation of KIAA0101 expression could affect the metastasis of EOC cells. We transfected KIAA0101 siRNA or control siRNA into SKOV3 and COV644 cells, and confirmed the downregulated expression of KIAA0101 in SKOV3 and COV644 cells after 48 h (Fig. 2a). We performed western blot to assess the expression of EMT markers, E-cadherin and N-cadherin. As shown in Fig. 2b, knockdown of KIAA0101 significantly increased E-cadherin and decreased N-cadherin expression. Furthermore, we discovered that in both cell lines, knockdown of KIAA0101 resulted in a significantly decrease in migration and invasion compared to those transfected with control siRNA, as determined by Transwell assays (Fig. 2c, d). Collectively, these results indicate that KIAA0101 may be required for the metastatic ability of EOC cells.

**Fig. 2:** Knockdown of KIAA0101 inhibits ovarian cancer cell migration and invasion. **a** Expression levels of KIAA0101 was determined by western blot in SKOV3 and COV644 cells transfected with KIAA0101 siRNA (siR-KIAA0101) or control siRNA (siR-Control). **b** Western blot analysis of E-cadherin and N-cadherin in SKOV3 and COV644 cells transfected with siR-KIAA0101 or siR-Control. **c** Migration and **d** Invasion assays in SKOV3 and COV644 cells transfected with siR-KIAA0101 or siR-Control. **p < 0.01, ***p < 0.001 compared with siR-Control transfected cells

### Knockdown of KIAA0101 inhibits EOC cell chemoresistance

KIAA0101 has been reported involving in drug resistance in esophageal and hepatocellular cancers [19, 24]. To explore whether KIAA0101 regulates EOC chemoresistance, we first treated SKOV3 and COV644 cells with 8 µM Cisplatin for 24 h and then changed to complete medium without Cisplatin for 48 h. KIAA0101 expression were examined at different time points. The results revealed that KIAA0101 was significantly upregulated after 6 h of Cisplatin treatment (Fig. 3a). We next treated EOC cells with different concentration of Cisplatin and performed MTT assays to examine cell growth rate. As shown in Fig. 3b, knockdown of KIAA0101 resulted in EOC cells more sensitive to Cisplatin treatment.

**Fig. 3:** Knockdown of KIAA0101 enhances ovarian cancer cell chemosensitivity. **a** SKOV3 and COV644 cells were cultured in complete medium with Cisplatin (8 µM) for 24 h, then medium was changed without Cisplatin for 48 h. The KIAA0101 expression were examined by qRT-PCR at different time points indicated. **b** MTT cell growth rate and **c** colony formation assays were performed in KIAA0101 knockdown SKOV3 and COV644 cells treated with different concentration of Cisplatin indicated. *p < 0.05 compared with siR-Control transfected cells

Additionally, colony formation assays demonstrated that knockdown of KIAA0101 significantly inhibited EOC cell growth with Cisplatin treatment (Fig. 3c). Collectively, these results indicated that KIAA0101 is essential for the resistance of EOC cell to Cisplatin.

### KIAA0101 regulates Wnt/β-catenin signaling in EOC cells

KIAA0101 regulates Wnt/β-catenin signaling in colon cancer cells [25]. In order to elucidate the molecular mechanisms of KIAA0101′s function in EOC, TOP flash reporter luciferase assays revealed the Wnt/β-catenin signaling activity was inhibited by depletion of KIAA0101 (Fig. 4a). We then examined β-catenin levels in the nucleus and cytoplasm of SKOV3 and COV644 cells in response to KIAA0101 silencing. The result showed that depletion of KIAA0101 inhibited β-catenin nuclear translocation (Fig. 4b). Furthermore, we performed qRT-PCR and western blot to investigate the expression of Wnt/β-catenin signaling downstream genes, Axin2 and c-myc. Consistently, the expression of Axin2 and c-myc was decreased after knockdown of KIAA0101 (Fig. 4c, d). These findings provided the evidences that KIAA0101 regulates Wnt/β-catenin signaling.

**Fig. 4:** KIAA0101 regulates Wnt/β-catenin signaling in EOC cells. **a** Luciferase activities in SKOV3 and COV644 cells 48 h after co-transfection with TOP flash luciferase plasmid and siR-KIAA0101 or siR-Control. **b** Levels of β-catenin was determined by Western blot in nucleus and cytoplasm of SKOV3 and COV644 cells transfected with siR-KIAA0101 or siR-Control. **c** mRNA and **d** protein levels of Axin2 and c-myc in SKOV3 and COV644 cells transfected with siR-KIAA0101 or siR-Control. *p < 0.05 compared with siR-Control transfected cells

### KIAA0101 is targeted by miR-429

We employed the bioinformatic Target Scan tools to predict the miRNA targeting KIAA0101, and found that miR-429 was one of the miRNA potentially binding KIAA0101 (Fig. 5a). MiR-429 plays an important role in EOC metastasis and chemoresistance. In order to validate that KIAA0101 was a direct target gene of miR-429, we constructed luciferase reporter plasmid with the wild type and mutant KIAA0101 3′-UTR region (Fig. 5b). We then co-transfected these plasmids into HEK293T cells with miR-429 and control miRNA, respectively. Results showed the transfection of miR-429 significantly reduced the luciferase activity of wild type KIAA0101 3′-UTR reporter, but not mutant KIAA0101 3′-UTR reporter (Fig. 5c). Consistently, miR-429 remarkably reduced KIAA0101 levels in SKOV3 and COV644 cells (Fig. 5d). Furthermore, we found an inverse correlation between the expression of KIAA0101 and miR-429 in 40 EOC tissue samples (Fig. 5e). Collectively, these results indicated that miR-429 inhibited the expression of KIAA0101 by targeting its 3′-UTR region.

**Fig. 5:** KIAA0101 is targeted by miR-429. **a** The putative binding sites of miR-429 on the KIAA0101 3′-UTR region. **b** Wild type (WT) of KIAA01013′-UTR region was mutated. **c** Luciferase activities in SKOV3 and COV644 cells 48 h after co-transfected with KIAA0101 3′-UTR wild type or mutant (Mut) luciferase plasmid and miR-429 or miR-Control. **p < 0.01 compared to miR-Control transfected cells. **d** Levels of KIAA0101 protein was determined by Western blot in SKOV3 and COV644 cells transfected with miR-429 or miR-Control. **e** The correlation of the expression levels of KIAA0101 and miR-429 in 40 EOC tissue samples (*r* = −0.648, *p* < 0.001)

### MiR-429 affected EOC cells partially through KIAA0101 mediated-Wnt/β-catenin signaling

Our previous results showed that downregulation of KIAA0101 inhibited EOC cell metastasis and Cisplatin chemoresistance, KIAA0101 regulates Wnt/β-catenin signaling and KIAA0101 was a target of miR-429. It is possible that miR-429 exerted its functions on EOC cells via KIAA0101 mediated-Wnt/β-catenin signaling pathway. If this is the case, then the relief of KIAA0101 suppression would reverse the regulation of miR-429 on EOC cells. To test this hypothesis, we simultaneously co-transfected plasmids encoding KIAA0101 into miR-429 overexpressing SKOV3 cells. These plasmids did not contain the 3′-UTR region of KIAA0101, and were therefore resistant to miR-429 regulation. We found that while overexpression of miR-429 reduced the expression of KIAA0101, but co-transfection of KIAA0101-overexpressing plasmids completely restored the levels of KIAA0101 protein as determined by Western blot analysis (Fig. 6a). In these cells, nuclear β-catenin levels and TOP flash luciferase activity inhibited by miR-429 overexpression were partially restored by KIAA0101 overexpression (Fig. 6b, c). The decreased expression of Axin2 and c-myc induced by miR-429 overexpression was partially abrogated by KIAA0101 overexpression (Fig. 6d, e). We then performed cell migration and invasion assays. As shown in Fig. 7a, b, transfection of KIAA0101-expressing plasmid partially reversed the inhibition of EOC cell metastasis (Fig. 7a, b). Furthermore, reduction of cell growth rate induced by miR-429 with Cisplatin treatment was partially restored by KIAA0101 (Fig. 7c). Together, these data suggested that miR-429 inhibited metastasis and chemoresistance of EOC cells, at least in part, via KIAA0101 mediated-Wnt/β-catenin signaling pathway.

**Fig. 6:** MiR-429 regulates Wnt/β-catenin signaling pathway partially through KIAA0101. **a** Levels of KIAA0101 protein was determined by Western blot in SKOV3 cells transfected with miR-429 or miR-Control, together with either vector control or plasmids encoding KIAA0101. **b** Levels of β-catenin was determined by Western blot in nucleus and cytoplasm of SKOV3 cells transfected with miR-429 or miR-Control, together with either vector control or plasmids encoding KIAA0101. **c** Luciferase activities in SKOV3 cells 48 h after transfection with miR-429 or miR-Control, together with either vector control or plasmids encoding KIAA0101. **d** mRNA and **e** protein levels of Axin2 and c-myc in SKOV3 cells transfected with miR-429 or miR-Control, together with either vector control or plasmids encoding KIAA0101. *p < 0.05 compared with siR-Control transfected cells

**Fig. 7:** MiR-429 affected EOC cells partially through KIAA0101. **a** Transwell migration assay and **b** Transwell invasion assays in SKOV3 cells transfected with either vector control or plasmids encoding KIAA0101. **c** MTT cell growth rate was performed in SKOV3 cells transfected with either vector control or plasmids encoding KIAA0101, when treated with Cisplatin (8 µM). *p < 0.05 compared with siR-Control transfected cells

## Discussion

In this study, we investigated the role of miR-429 and its target gene KIAA0101 in regulation of migration and chemoresistance of EOC cell lines, SKOV3 and COV644. We found that expression of KIAA0101 was elevated in the metastatic EOC tissues, compared to primary EOC tissue. Ectopic overexpression of miR-429 showed similar inhibitory effects as siRNA-mediated depletion of KIAA0101 on migration and chemoresistance of EOC cells. Mechanistically, we found this inhibitory effects were mediated by Wnt/β-catenin signaling pathway. Overexpression of miR-429 and depletion of KIAA0101 significantly suppressed the translocation of β-catenin into nucleus.

To our knowledge, this is the first time that we have demonstrated KIAA0101 inhibited invasion and resistance to Cisplatin treatment of EOC cells by enhancing Wnt/β-catenin signaling. KIAA0101 was initially identified by the associate factor of PCNA, which is essential for the proliferation of normal cells and tumor cells [26]. Recent studies have shown the KIAA0101 may serve as a biomarker for poor prognosis and recurrence in multiple human cancers [18, 27]. In this study, we furthered revealed that KIAA0101 was also necessary for the migration activity and chemoresistance of EOC cells, which is mediated by Wnt/β-catenin signaling. Wnt/β-catenin signaling was reported to play a critical role in ovarian tumorigenesis and progression by driving epithelial-to-mesenchymal transition (EMT) [28, 29]. In ovarian cancer, Wnt/β-catenin signaling might be activated by increased expression of β-catenin and glycogen synthase kinase 3β (GSK3β), mutations of catenin beta 1 (CTNNB1) gene, and so on [30, 31]. A recent study has also revealed that Wnt/β-catenin signaling maintains stem-like properties and promotes resistance to Cisplatin and Platinum in high-grade SOC cells [32]. Given the role of the Wnt/β-catenin signaling, specific Wnt/β-catenin signaling inhibitors have generated a great amount of enthusiasm in treatment for ovarian cancer [28]. Thus, our findings suggest that KIAA0101 may represent a promising therapeutic target of EOC. However, the mechanism by which KIAA0101 regulates Wnt/β-catenin signaling activity remains to be investigated.

We also found KIAA0101 was directly regulated by miR-429. We firstly employed the bioinformatic Target Scan tools to predict the miRNA targeting KIAA0101, and the binding of miR-429 to the 3′ UTR of KIAA0101 mRNA was further confirmed by luciferase assay. However, it is worthy to note that miRNA usually have multiple targets [33, 34]. In this study, co-transfection of KIAA0101 in miR-429 overexpressed EOC cells did not fully abrogate the effect of miR-429 overexpression, indicating other factors may be involved in this process. Further studies are with required to identify other targets of miR-429 in EOC cells that regulate the process of malignancy. Furthermore, miR-429 was found to be downregulated in several human cancers [12, 13, 35], but upregulation of miR-429 was negatively correlated to prognosis of patients with SOC [16], indicating different role of miR-429 in regulating cancer progression that are initiated from different tissues. In this study, we reported the role of miR-429 in regulation of chemoresistance of EOC cells for the first time. The role of miR-429 in regulation of chemoresistance in other cancers may be investigated in the future.

## Conclusions

KIAA0101, targeted by miR-429, promotes invasion and chemoresistance of EOC cells through Wnt/β-catenin signaling pathway. Both miR-429 and KIAA0101 may be used to predict the prognosis of patients with EOCs, and may represent new therapeutic targets of EOCs. However, more investigation needs to be carried out to investigate how KIAA0101 regulates Wnt/β-catenin signaling, and whether targeting miR-429 and/or KIAA0101 is capable of suppress EOC progression in vivo.

## Abbreviations

EOC: epithelial ovarian cancer
miRNA: microRNA
MPO: myeloperoxidase
SOC: serous ovarian carcinoma
PCNA: proliferating cell nuclear antigen
p15PAF: PCNA-associate factor
EMT: epithelial-to-mesenchymal transition
GSK3β: glycogen synthase kinase 3β
CTNNB1: catenin beta 1

## References

[1] McGuire V, Jesser CA, Whittemore AS (2002). Survival among US women with invasive epithelial ovarian cancer. Gynecol Oncol.

[2] Quirk JT, Natarajan N (2005). Ovarian cancer incidence in the United States, 1992–1999. Gynecol Oncol.

[3] Morgan RJ, Alvarez RD, Armstrong DK, Boston B, Burger RA, Chen LM, Copeland L, Crispens MA, Gershenson D, Gray HJ (2011). Epithelial ovarian cancer. J Natl Compr Canc Netw.

[4] Lengyel E (2010). Ovarian cancer development and metastasis. Am J Pathol.

[5] Chen J, Wang L, Matyunina LV, Hill CG, McDonald JF (2011). Overexpression of miR-429 induces mesenchymal-to-epithelial transition (MET) in metastatic ovarian cancer cells. Gynecol Oncol.

[6] Matei DE, Nephew KP (2010). Epigenetic therapies for chemoresensitization of epithelial ovarian cancer. Gynecol Oncol.

[7] Harries M, Gore M (2002). Part I: chemotherapy for epithelial ovarian cancer–treatment at first diagnosis. Lancet Oncol.

[8] Winter J, Jung S, Keller S, Gregory RI, Diederichs S (2009). Many roads to maturity: microRNA biogenesis pathways and their regulation. Nat Cell Biol.

[9] Osada H, Takahashi T (2007). MicroRNAs in biological processes and carcinogenesis. Carcinogenesis.

[10] Mirnezami A, Pickard K, Zhang L, Primrose J, Packham G (2009). MicroRNAs: key players in carcinogenesis and novel therapeutic targets. Eur J Surg Oncol.

[11] Zhang M, Dong BB, Lu M, Zheng MJ, Chen H, Ding JZ, Xu AM, Xu YH (2016). miR-429 functions as a tumor suppressor by targeting FSCN1 in gastric cancer cells. Onco Targets Ther.

[12] Sun Y, Shen S, Liu X, Tang H, Wang Z, Yu Z, Li X, Wu M (2014). MiR-429 inhibits cells growth and invasion and regulates EMT-related marker genes by targeting Onecut2 in colorectal carcinoma. Mol Cell Biochem.

[13] Ye ZB, Ma G, Zhao YH, Xiao Y, Zhan Y, Jing C, Gao K, Liu ZH, Yu SJ (2015). miR-429 inhibits migration and invasion of breast cancer cells in vitro. Int J Oncol.

[14] Park SM, Gaur AB, Lengyel E, Peter ME (2008). The miR-200 family determines the epithelial phenotype of cancer cells by targeting the E-cadherin repressors ZEB1 and ZEB2. Genes Dev.

[15] Nam EJ, Yoon H, Kim SW, Kim H, Kim YT, Kim JH, Kim JW, Kim S (2008). MicroRNA expression profiles in serous ovarian carcinoma. Clin Cancer Res.

[16] Hu X, Macdonald DM, Huettner PC, Feng Z, El Naqa IM, Schwarz JK, Mutch DG, Grigsby PW, Powell SN, Wang X (2009). A miR-200 microRNA cluster as prognostic marker in advanced ovarian cancer. Gynecol Oncol.

[17] Zhao H, Lo YH, Ma L, Waltz SE, Gray JK, Hung MC, Wang SC (2011). Targeting tyrosine phosphorylation of PCNA inhibits prostate cancer growth. Mol Cancer Ther.

[18] Kato T, Daigo Y, Aragaki M, Ishikawa K, Sato M, Kaji M (2012). Overexpression of KIAA0101 predicts poor prognosis in primary lung cancer patients. Lung Cancer.

[19] Cheng Y, Li K, Diao D, Zhu K, Shi L, Zhang H, Yuan D, Guo Q, Wu X, Liu D (2013). Expression of KIAA0101 protein is associated with poor survival of esophageal cancer patients and resistance to cisplatin treatment in vitro. Lab Invest.

[20] Zhu K, Diao D, Dang C, Shi L, Wang J, Yan R, Yuan D, Li K (2013). Elevated KIAA0101 expression is a marker of recurrence in human gastric cancer. Cancer Sci.

[21] Jain M, Zhang L, Patterson EE, Kebebew E (2011). KIAA0101 is overexpressed, and promotes growth and invasion in adrenal cancer. PLoS One.

[22] Xia B, Li H, Yang S, Liu T, Lou G (2016). MiR-381 inhibits epithelial ovarian cancer malignancy via YY1 suppression. Tumour Biol..

[23] Xia B, Yang S, Liu T, Lou G (2015). miR-211 suppresses epithelial ovarian cancer proliferation and cell-cycle progression by targeting cyclin D1 and CDK6. Mol Cancer.

[24] Liu L, Chen X, Xie S, Zhang C, Qiu Z, Zhu F (2012). Variant 1 of KIAA0101, overexpressed in hepatocellular carcinoma, prevents doxorubicin-induced apoptosis by inhibiting p53 activation. Hepatology.

[25] Jung HY, Jun S, Lee M, Kim HC, Wang X, Ji H, McCrea PD, Park JI (2013). PAF and EZH2 induce Wnt/beta-catenin signaling hyperactivation. Mol Cell.

[26] Yu P, Huang B, Shen M, Lau C, Chan E, Michel J, Xiong Y, Payan DG, Luo Y (2001). p15^ P^ A^ F, a novel PCNA associated factor with increased expression in tumor tissues. Oncogene.

[27] Hosokawa M, Takehara A, Matsuda K, Eguchi H, Ohigashi H, Ishikawa O, Shinomura Y, Imai K, Nakamura Y, Nakagawa H (2007). Oncogenic role of KIAA0101 interacting with proliferating cell nuclear antigen in pancreatic cancer. Cancer Res.

[28] Gatcliffe TA, Monk BJ, Planutis K, Holcombe RF (2008). Wnt signaling in ovarian tumorigenesis. Int J Gynecol Cancer.

[29] Hou M, Cheng Z, Shen H, He S, Li Y, Pan Y, Feng C, Chen X, Zhang Y, Lin M (2015). High expression of CTHRC1 promotes EMT of epithelial ovarian cancer (EOC) and is associated with poor prognosis. Oncotarget.

[30] Rask K, Nilsson A, Brännström M, Carlsson P, Hellberg P, Janson PO, Hedin L, Sundfeldt K (2003). Wnt-signalling pathway in ovarian epithelial tumours: increased expression of β-catenin and GSK3β. Br J Cancer.

[31] Gamallo C, Palacios J, Moreno G, de Mora JC, Suárez A, Armas A (1999). β-catenin expression pattern in stage I and II ovarian carcinomas: relationship with β-catenin gene mutations, clinicopathological features, and clinical outcome. Am J Pathol.

[32] Nagaraj AB, Joseph P, Kovalenko O, Singh S, Armstrong A, Redline R, Resnick K, Zanotti K, Waggoner S, DiFeo A (2015). Critical role of Wnt/beta-catenin signaling in driving epithelial ovarian cancer platinum resistance. Oncotarget.

[33] Bartel DP (2009). MicroRNAs: target recognition and regulatory functions. Cell.

[34] Croce CM (2009). Causes and consequences of microRNA dysregulation in cancer. Nat Rev Genet.

[35] Li J, Du L, Yang Y, Wang C, Liu H, Wang L, Zhang X, Li W, Zheng G, Dong Z (2013). MiR-429 is an independent prognostic factor in colorectal cancer and exerts its anti-apoptotic function by targeting SOX2. Cancer Lett.

